RETRACTED

# Alpha Protein Kinase 2 Promotes Esophageal Cancer via Integrin Alpha 11

**DOI:** 10.1155/2022/7676582

**Published:** 2022-06-29

**Authors:** Julaiti Ainiwaer, Liwei Zhang, Maidiniyeti Niyazi, Edris Awut, Shutao Zheng, Ilyar Sheyhidin, JiangHong Dai

**Affiliations:** ^1^School of Public Health, Xinjiang Medical University, China; ^2^Department of Thoracic Surgery, First Affiliated Hospital of Xinjiang Medical University, China; ^3^The Clinical Medicine Research Institute, First Affiliated Hospital of Xinjiang Medical University, China

## Abstract

**Background:**

As a common disease around the world, esophageal cancer (EC) primarily includes two subclasses: esophageal adenocarcinoma and esophageal squamous cell carcinoma. Mortality has been rising over the years; hence, exploring the mechanism of EC development has become critical. Among the alpha protein kinases, alpha protein kinase 2 (ALPK2) presumably has a connection with EC, but it has never been revealed before.

**Methods:**

In this study, IHC analysis was used for ALPK2 expression quantification in ES tissues. TE-1 and Eca-109, which are both human EC cell lines, were used for *in vitro* analysis of cell proliferation, migration, apoptosis, and colony formation.

**Results:**

ALPK2 was found to have an abundant expression within EC tissues (*P* < 0.001), as well as in the two selected human EC cell lines (*P* < 0.05). The data showed that ALPK2 depletion suppressed EC cell proliferation, migration, and colony formation, meanwhile stimulating apoptosis (*P* < 0.001). The *in vivo* experiments also displayed inhibitory effects caused by ALPK2 depletion on EC tumorigenesis (*P* < 0.001). It was further validated that ALPK2 depletion made the phosphorylation of Akt and mTOR, as well as CDK6 and PIK3CA levels downregulated (*P* < 0.001). Mechanistically, we identified integrin alpha 11 (ITGA11) as a downstream gene of ALPK2 regulating EC. More importantly, we found that ITGA11 elevation promoted cell proliferation and migration and rescued the suppression effects caused by ALPK2 depletion (*P* < 0.001).

**Conclusions:**

ALPK2 promotes esophageal cancer via integrin its downstream gene alpha 11; ALPK2 can potentially act as a target for the treatment of EC.

## 1. Introduction

Esophageal cancer (EC), which includes esophageal adenocarcinoma (EAC) and esophageal squamous cell carcinoma (ESCC) [1], is an extremely aggressive disease that affects patients worldwide and lies sixth most common cause of cancer death [2]. Over the years, the incidence of EC is sharply increased, thus posing a major challenge to global health. Surgical resection, chemotherapy, and radiotherapy are the initial clinical strategies currently employed for the treatment of EC. In spite of tremendous efforts and advances made in treating EC, the mortality is alarming owing to the inadequate efficacy and harmful side effects of conventionally employed treatment strategies [3]. Targeted therapies, as a newly developed technique, have been verified to perform key functions in the treatment of EC [4]. Taking bevacizumab and cetuximab as examples, they make the treatment outcome better to a certain degree via targeting vascular endothelial growth factor (VEGF) and epidermal growth factor receptor (EGFR), respectively [5]. Nevertheless, some disadvantages of the therapy follow. For instance, the life of patients can be prolonged by targeted therapy, but they do not recover fully because of drug resistance. It is therefore essential to seek more effective targets for EC therapy, and the understanding of mechanism associated with the development of this lethal illness becomes crucial.

RETRACTED

A member of the alpha kinase family, alpha protein kinase 2 (ALPK2), has a largely conserved alpha protein kinase domain. Initially, a domain of ALPK2 is identified to be similar to that of the elongation factor 2 kinase and is housed at 18q21.31 [6, 7]. ALPK2 has been considered to be a Wnt/*β*-catenin signaling pathway inhibitor and a regulator for cardiac development [8]. It has been reported in the literature that ALPK2 worked as a potential promotor for the metastasis and development of renal cell carcinoma [9]. ALPK2 was also found to exert a cancer-promoting role in carcinogenic process of bladder cancer by regulating DEPDC1A, a newly discovered tumor-related gene which was reported to be overexpressed in malignant tumors such as bladder cancer, breast cancer, and lung adenocarcinoma [10]. Furthermore, abnormal expression of ALPK2 could hasten proliferation, migration, and restraint apoptosis of ovarian cancer cells via affecting EMT-related proteins as well as the regulation of downstream pathways [11]. However, there is only limited literature discussing the role of ALPK2 and the function of ALPK2 in EC remains majorly unknown.

This study was aimed at investigating the roles of ALPK2 in EC development and progression and exploring the effect of ALPK2 expression on proliferation, migration, apoptosis, colony formation, and tumorigenesis of esophageal carcinoma cells and tissues in vitro and in vivo, furthermore revealing the regulatory mechanism of ALPK2 on PI3K/AKT/mTOR signaling pathways and its upstream and downstream genes, intending to evaluate the effects of ALPK2 depletion on EC cell phenotypes.

## 2. Materials and Methods

### 2.1. Cell Culture

TE-1 and Eca-109 cells were provided by Cell Resource Center, Institute of Basic Medicine, Chinese Academy of Medical Sciences (Beijing, China). Cell culture was carried out in a 1640 medium containing 10% FBS, followed by incubation with 5% CO_2_ in a 37°C incubator. We performed cell line authentication at the beginning of the experiment and repeated every two months, by short tandem repeat (STR) analysis.

RETRACTED

### 2.2. Immunohistochemistry (IHC)

157 esophageal cancer and 38 paracarcinoma tissue microarray chips (#ES2001a) were provided by Xi'an Alina Biotechnology Co., Ltd. (Xian, China). Individual patients consented and furnished the pertinent clinical characteristics. ALPK2 antibody (1 : 100, Biorbyt, #orb314576) and secondary antibody were provided by Wuhan Booute Biotechnology Co., Ltd. (Wuhan, China). The expression of ALPK2 protein was assessed using immunohistochemical methods. Analysis of the photos was made taking into view the IHC scoring standard comprising four classes: +++ positive (9-12), ++ positive (5-8), positive (1-4), and negative (0), according to the product of the intensity of staining (varying from weak to strong) as well as staining extent scores; the grading for which follows the below sequence as 0 (0%), 1 (1-25%), 2 (26-50%), 3 (51-75%), or 4 (76-100%) [12].

### 2.3. Plasmid Construction, Lentivirus Infection

Shanghai Bioscienceres Co., Ltd. (Shanghai, China) designed three corresponding RNAi target sequences (from 5′ to 3′: GCGAAGACCTTGGCATTTATT, TGCTAATAATGAGTGCTTTCA, ACAGTCCAGAGGATGCTGAGT) using ALPK2 as templates. In addition, we overexpressed ITGA11 using LV-013-ITGA11 Plasmid (Shanghai Bioscienceres Co., Ltd.). Insertion of The ITGA11 and ALPK2 target sequences was made into the BR-V-108 vector at both ends via the restriction sites followed by subsequent transformation into TOP 10 E. coli competent cells (Tiangen, Beijing, China). PCR identification was employed for screening the positive recombinants, and the EndoFree maxi plasmid kit (Tiangen, Beijing, China) was employed for the extraction of plasmid following the instructions detailed by the manufacturer. The qualified plasmids were shifted to downstream platforms for lentivirus packaging. A coinfection system based on three-plasmid BR-V112 BR-V307 and BR-V108 was employed for collecting the 239T cell supernatant at 48 h and 72 h following infection, and the lentivirus quality was assessed. Ultimately, 20 *μ*L 1 × 10^8^ TU/mL lentivirus was added to infect Eca-109/TE-1 cells lying in the logarithmic growth phase, followed by culture in 1640 medium in a 6-well dish, with 10% FBS at a density of 2 × 10^5^ cells per well. Microscopic fluorescence, qPCR, and western blot were carried out to assess the knockdown efficiency and cell infection efficiency.

RETRACTED

### 2.4. RNA Extraction and qRT-PCR

Isolation of the total RNA was carried out following the protocol outlined by the manufacturer of TRIzol reagent (Sigma, St. Louis, MO, USA). Using the Promega M-MLV Kit (Promega Corporation, Madison, Wisconsin, USA), RNA was reversely transcribed to cDNA. The qRT-PCR system was 10 *μ*L based on SYBR Green Master Mix Kit (Vazyme, Nanjing, Jiangsu, China), and the relative expression of mRNA was analyzed by the 2^-△△Ct^ method. qPCR employed the sequences of the following primers (5′-3′). The forward and reverse primers of ALPK2 were TCCGAAGGACCAGGGACTCTAT and CGGTGAACCCCTTCTCCAAA (from 5′ to 3′). The corresponding primers of GAPDH were TGACTTCAACAGCGACACCCA and CACCCTGTTGCTGTAGCCAAA.

### 2.5. Western Blot Assay

TE-1 and Eca-109 cells after infection were gathered and subjected to lysis using 1× Lysis Buffer (Cell Signal Technology, Danvers, MA). Additionally, extraction of total proteins was attempted using 10% SDS-PAGE which were then shifted onto PVDF membranes and blocked with TBST solution comprising 5% skim milk. The membranes were subsequently incubated with the primary and secondary antibodies for 2 h, following which a solution of TBST was used to wash the membranes thrice. Ultimately, color was rendered using the ECL+ Plus™ western blotting system kit and X-ray imaging was carried out. Western blot employed the following primary antibodies: ALPK2 (1 : 1000, Abcam, #ab111909), GAPDH (1 : 3000, Bioworld, #AP0063), Akt (1 : 1000, CST, #4685), P-Akt (1 : 500, systems, #AF887-sp), mTOR (1 : 3000, CST, #2972), P-mTOR (1 : 1000, Beijing Solebold Antibody, #K006205P), CDK6 (1 : 1000, Abcam, #ab151247), and PIK3CA (1 : 1000, Abcam, #ab40776). Goat Anti-Rabbit (1 : 3000, Beyotime, #A0208) was the secondary antibody used in western blot analysis.

### 2.6. MTT Assay

Infected TE-1 and Eca-109 cells were digested and allowed to resuspend in the cell suspension at a density of 2000 cells/well. For 5 days, a 100 *μ*L cell suspension was grown in 96-well plates. Each well was repeated three times. 100 *μ*L DMSO and 20 *μ*L MTT (5 mg/mL) were added in the corresponding wells. A microplate reader (Tecan Infinite, Mannedorf Zurich, Switzerland) was used to determine the value of the optical density (OD) at a wavelength of 490 nm.

### 2.7. Celigo Cell Counting Assay

Upon the achievement of 70 to 90% confluence, the infected TE-1 and Eca-109 cells were plated into 96-well plates at a density of 2000 cells per well and housed in a 37°C incubator in a 5% CO_2_ atmosphere. A continuous 5-day cell proliferation curve was generated using images taken with a Celigo imaging cytometer (Nexcelom Bioscience, Lawrence, MA, USA).

RETRACTED

### 2.8. Cell Migration Assay

TE-1 cells and Eca-109 were infected and harvested and planted within a 96-well plate at a density of 5 × 10^4^ cells/well. Following that, the cells were placed in a 37°C incubator in a 5% CO_2_ atmosphere. A microscope was used to observe and photograph the cells at 4 h, 5 h, 24 h, and 48 h. This procedure was done three times, and cellular migration rate was assessed through these scratch images.

For the transwell test, the lentivirus-infected TE-1 and Eca-109 cells were cultured at a density of 8 × 10^4^ cells/mL followed by their loading into the top chamber comprising serum-free media. The top compartment was then moved to the bottom chamber and then inoculated for 48 hours with media containing 30% FBS. After that, cells were stained by 400 *μ*L of Giemsa, and the cellular migration level was measured.

### 2.9. Colony Formation Assay

TE-1 and Eca-109 cells were digested and resuspended for seeding into a 6-well plate at a density of 2 mL/well to grow eight days, and the media was changed every three days. A fluorescent microscope (Olympus, Tokyo, Japan) was employed for recording the visible clones. Subsequently, the cells were rinsed in PBS. Then, 1 mL 4% paraformaldehyde was then used for fixation, and 500 mL Giemsa (Dingguo, Shanghai, China) was used for staining. Subsequently, the colonies were counted.

### 2.10. Cell Apoptosis Assay

TE-1 and Eca-109 cells infected with lentivirus were grown in 6-well plates (each well containing 2 mL) for 5 days. Then, Annexin V-APC (10 *μ*L) was added for staining in the dark at room temperature for 10-15 minutes. FACSCalibur (BD Biosciences, San Jose, CA, USA) was utilized for determining the amount of cellular apoptosis.

### 2.11. Human Apoptosis Antibody Array

Following cell lysis, the blocking of the handling array membranes was carried out with 2 mL 1Wash Buffer II and allowed to incubate with 1Biotin-conjugated anticytokines and cell lysates overnight at a temperature of 4°C. Finally, a chemiluminescence imaging device was used to track membrane signals.

### 2.12. Nude Mouse Model Assay

Subcutaneous injection of Eca-109 cells infected with shCtrl and shALPK2 into four-week-old female BALB-c nude mice (*n* = 10 for individual groups) yielded the xenograft models. The tumor volume was assessed during the feeding phase. After 59 feeding days, intraperitoneal injection of 0.7% sodium pentobarbital was given for a few minutes, and the fluorescence was recorded using *in vivo* imaging equipment (IVIS Spectrum, PerkinElmer). Then, the scarification of the mice was carried out via the method of cervical dislocation. The tumors were removed for weighing and photography. The First Affiliated Hospital of Xinjiang Medical University's Ethics Committee approved the study design.

RETRACTED

### 2.13. Ki-67 Staining

4% paraformaldehyde and 0.3% Triton X-100 were used to fix slices of mouse tumor tissues. The primary antibody Ki-67 (1 : 300, Abcam, Ab16667) was added to the slides which were incubated with it in the dark at 4°C overnight. The secondary antibody goat anti-rabbit IgG H&L (HRP) (1 : 400, Abcam, Ab97080) was introduced in the same manner. Ultimately, eosin and hematoxylin (Baso, Zhuhai, Guangdong, China) were used to stain the slides, which were then examined under a microscope.

### 2.14. Statistical Analysis

SPSS 19.0 (IBM, SPSS, Chicago, IL, USA) and GraphPad Prism 8 (San Diego, CA, USA) were used for the analysis of the data, and the results were given as the mean ± SD (standard deviation). The statistical significance was ascertained by making use of the Student *t*-test and one-way ANOVA. The link between ALPK2 expression and esophageal cancer patient characteristics was assessed using Spearman correlation analysis and Mann–Whitney *U* analysis. *P* < 0.05 was regarded to be a statistically significant difference. All of the tests were carried out thrice.

## 3. Results

### 3.1. ALPK2 Displayed Upregulated Expression in Esophageal Cancer

To analyze the expression patterns of ALPK2, we first compared the matched paracarcinoma tissue and esophageal cancer microarrays, providing a valuable result of ALPK2 upregulation in EC tissues (*P* < 0.001, Table 1, Figure 1(a)). Additionally, in a panel of human EC cell lines analyzed, ALPK2 expression appeared to be relatively higher in TE-1 cells and Eca-109 (*P* < 0.05, Figure 1(b)). The results from the Mann–Whitney *U* analysis identified that ALPK2 expression was closely linked to pathological stage and tumor lymphatic metastasis (*P* < 0.05, Table 2). In Spearman analysis, we observed a positive relationship between ALPK2 expression with pathological stage and lymphatic metastasis (correlation of 0.203 and 0.206, respectively) (*P* < 0.05, Table 3). It can be concluded from the results that ALPK2 might cross the entire development and progression of EC.

### 3.2. Development of ALPK2 Knockdown Cell Models

Next, we sought to build up TE-1 and Eca-109 cell models for subsequent use in the experiments to study mechanism. To test whether lentivirus plasmids were successfully established, we infected Eca-119 cells with three lentivirus plasmids (shALPK2-1, shALPK2-2, and shALPK2-3), finding that the knockdown efficiency of ALPK2 in the shALPK2-1 group was 74.1% (*P* < 0.05, Figure 1(c)). As a result, shALPK2-1 was selected for following cell model construction. For this analysis, the green fluorescent protein (GFP) inside TE-1 and Eca-109 cells demonstrated >80% efficiency of infection (Figure 1(d)). Next, we determined ALPK2 expression levels in shALPK2 Eca-109 and TE-1 cells through western blot and qRT-PCR analysis. In both these analyses, ALPK2 expression was significantly decreased relative to ALPK2 levels in the corresponding shCtrl cells (Figures 1(e) and 1(f)). Cumulatively, several lines of evidence indicated that ALPK2 knockdown cell models were better constructed.

RETRACTED

### 3.3. ALPK2 Depletion Weakened the Migration and Proliferation of Esophageal Cancer Cells, Ameliorated Cell Apoptosis *In Vitro*

Following shALPK2-1 infection, our analysis of cell phenotypes in TE-1 and Eca-109 cellular models demonstrated that there was a strong inhibition in the degree of cell proliferation in shALPK2 cells in comparison to shCtrl cells (*P* < 0.001, Figure 2(a)). The phenomenon of suppressed migration simultaneously occurred in shALPK2 TE-1 and Eca-109 cells via both transwell and wound-healing assays (*P* < 0.001, Figures 2(b) and 2(c)). In addition, as depicted in the resulting colony formation assay, this was consistent with our prediction that the ability of colony formation in shALPK2 cell models was attenuated (*P* < 0.001, Figure 2(d)). An idea supported by *in vitro* studies demonstrated that ALPK2 depletion could promote EC cell apoptosis (*P* < 0.001, Figure 3(a)). Next, some apoptosis-related elements were evaluated, accompanying by the upregulation of DR6, BIM, CD40L, cytoC, Fas, HSP60, FasL, IGFBP-3, IGFBP-4, IGFBP-5, IGFBP-6, p21, and p27 (Figures 3(b)–3(d)). On the basis of these strong evidences, we concluded that the migration and cell proliferation capabilities were all weakened because of ALPK2 depletion, while accelerating their apoptosis.

### 3.4. ALPK2 Depletion Curbed Esophageal Cancer Tumorigenesis *In Vivo*

In this section, we focused here on esophageal cancer tumorigenesis upon silencing ALPK2. Subcutaneous injection of shALPK2 Eca-109 cells was given to the nude mice for establishing subcutaneous xenograft models (Figure 4(a)). Specifically, the volume and weight of transplanted tumors displayed an apparent reduction when compared to the shCtrl group (*P* < 0.001, Figures 4(b)–4(d)). The results of *in vivo* imaging revealed a decreased fluorescence, which would be regarded as impaired tumor growth within the shALPK2 group (*P* < 0.001, Figure 4(e)). At the same time, we analyzed the level of proliferation marker Ki-67, which revealed that Ki-67 was largely suppressed in the absence of ALPK2 (Figure 4(f)). It should also be noted that cancer-related factors such as P-mTOR, CDK6, PIK3CA, and P-AKT were markedly downregulated (Figure 4(g)). Overall, these observations led to proposals that ALPK2 downregulation could be a causal event in inhibiting tumorigenesis of EC.

RETRACTED

### 3.5. ALPK2 Depletion Impaired Esophageal Cancer Development via the Downregulation of ITGA11

Finally, we investigated the mechanism behind ALPK2 regulating esophageal cancer. Through analyzing the Coexpedia website (https://www.coexpedia.org/hs_single.php?gene=ALPK2), we predicted the coexpressed genes of ALPK2, among which the top three were PAPPA, ITGA11, and RAB31 (Figure 5(a)). Subsequently, we assessed PAPPA, ITGA11, and RAB31 levels in ESCA samples from TCGA database using the UALCAN website (http://ualcan.path.uab.edu/cgi-bin/ualcan-res.pl), following that they were elevated in tumor tissues (*P* < 0.001, Figure 5(b)). Besides, employing ENCORI website (https://starbase.sysu.edu.cn/panGeneCoExp.php), the association between the above three and the expression level of ALPK2 was also constructed, indicating that they had a strong positive correlation with ALPK2 (Figure 5(c)). Next, we knocked down PAPPA, ITGA11, and RAB31 expression in Eca-109 cells using short hairpin RNA against PAPPA, ITGA11, and RAB31 mRNA (shPAPPA, shITGA11, and shRAB31) and negative control (shCtrl). In Celigo cell counting assay, we found that only silencing ITGA11 dramatically attenuated the ability of Eca-109 cell proliferation (*P* < 0.01, Figure 5(d)). We therefore selected ITGA11 for further investigation. With the purpose of identifying that the tumor suppressor effects of ALPK2 loss were mediated by ITGA11, we constructed TE-1 and Eca-109 cell models having ITGA11 overexpression and/or ALPK2 downregulation and tested cell phenotypes. Consistent with previous data, merely silencing ALPK2 inhibited TE-1 and Eca-109 cell proliferation and migration. On the other hand, the data of cell viability and migration detection showed that ITGA11 elevation led to increased cell viability and migration and rescued the suppression effects caused by ALPK2 depletion (Figures 5(e) and 5(f)), implying that ITGA11 has an indispensable part in ALPK2 inducing the cell viability and migration of TE-1 and Eca-109.

## 4. Discussion

EC is one of the top ten deadly cancers worldwide with its extremely high aggressiveness and poor survival rate [13], and only 20% of EC patients can be treated with surgery [14]. Other clinical methods for EC include radiotherapy and chemotherapy. However, mounting clinical trials showed that conventional chemotherapy drugs have limited efficacy and severe side effects [15]. Currently, the study on related targeted drugs for EC treatment still arouses general interest. Targeted therapy can improve the treatment outcome, but patients often face the emergence of drug resistance [4, 5]. Clearly, there is an urgent need to discover better and newer therapeutic techniques with improved efficacy and limited adverse impact against EC.

RETRACTED

ALPK2, an atypical alpha protein kinase, possesses a key role in human pluripotent stem cell development and zebrafish cardiogenesis by inhibiting the Wnt/-catenin signaling pathway [8]. ALPK2 has been linked to the development of colorectal cancer in a number of studies. ALPK2 regulates luminal apoptosis and the production of DNA repair-related genes, which is important in the shift of normal colonic crypt to adenoma [16]. Furthermore, earlier research has indicated a link between ALPK2 germline mutations and colorectal cancer in a number of instances [17]. With the exception of colorectal cancer, the link between ALPK2 and the majority of other human carcinomas is unknown. The current investigation revealed that the expression of ALPK2 had undergone upregulation in EC tissues relative to normal tissues and that it was significantly abundant in EC cell lines. ALPK2 deletion could dramatically limit the capability of EC cells to proliferate and create colonies. The data from the transwell and wound-healing experiments that followed showed that ALPK2 knockdown inhibited EC cell migration. On the other side, we discovered that knocking down ALPK2 promotes EC cell death by upregulation of apoptosis-related proteins such as p21, p27, BIM, cytoC, CD40L, DR6, Fas, FasL, HSP60, IGFBP-3, IGFBP-4, IGFBP-5, and IGFBP-6. More notably, the capacity of ALPK2 knockdown to inhibit tumor growth in mouse xenograft models was also demonstrated. ALPK2 was discovered to be a tumor promotor for EC in this investigation.

ITGA11, belonging to the integrin family, was identified as a downstream gene of ALPK2 that regulates EC. Integrins are heterodimers resulting from two types of subunits, the *α* (120-185 kD) and *β* (90-110 kD) subunits, which regulate the relationship of cells with their external environment [18]. In effect, these heterodimers are transmembrane receptors [19]. ITGA11 regulates collagen-mediated biological activities in cells, including cell migration, collagen recombination, and collagen deposition [20]. Furthermore, ITGA11 has been linked to the advancement of a number of malignancies. ITGA11 expression, for example, is significantly higher in individuals with NSCLC and is linked to poor overall survival [21]. ITGA11 has an extensive expression in esophageal squamous cell carcinoma and is linked to tumor cell migration and invasion, according to Chai et al. [22]. We discovered that increasing ITGA11 increased cell proliferation and migration, meanwhile rescuing the suppressive effects produced by ALPK2 depletion, indicating that ITGA11 is a mediator in ALPK2 EC regulation.

RETRACTED

Cell metabolism, growth, proliferation, and survival are all regulated by Akt (referred to as protein kinase B (PKB)) [23, 24]. We discovered that ALPK2 knockdown reduced the level of Akt phosphorylation. The serine/threonine-protein kinase mammalian target of rapamycin (mTOR) regulates cap-dependent translation, ribosomal protein translation, and protein synthesis. Tumorigenesis, angiogenesis, cell proliferation, and metastasis are all aided by abnormal mTOR signaling [25]. There are additional published articles stating that the mTOR pathway is abnormally activated in most ESCC cells, that high levels of P-mTOR are linked to poor ESCC prognosis, and that it is, therefore, a therapeutic target for ESCC [26, 27]. P-mTOR was similarly found to be downregulated when ALPK2 was depleted. CDK6 is a key regulator of cell cycle and proliferation [28] and has links with numerous areas of cancer research and prognosis [29]. Our findings consistently revealed that ALPK2 depletion resulted in considerable downregulation of CDK6, showing that ALPK2 depletion may be a mechanism for EC. PIK3CA, which encodes the PI3K catalytic subunit p110a and has been linked to a variety of human malignancies [30–32], was likewise shown to be downregulated when ALPK2 was silenced. Despite these findings, the precise mechanism of ALPK2's regulatory influence upon the formation and progression of EC remains unknown, and this will be the subject of future research.

In conclusion, our findings offered a critical framework for understanding the functions of ALPK2 in EC progression, highlighted the unique roles of ALPK2 depletion in EC cell morphologies, and speculated on ALPK2's antiesophageal cancer mechanism. These findings revealed fresh information about ALPK2's anticancer function and suggested that ALPK2 could be used to control EC.

## Figures and Tables

**Figure 1:** ALPK2 was upregulated in esophageal cancer, and ALPK2 depletion cell model was constructed. (a) ALPK2 expression in paracarcinoma tissues and esophageal cancer tissues was ascertained by IHC staining (ALPK2 expression in cells marked by arrows). (b) The levels of expression ALPK2 in esophageal cancer cell lines were determined by qRT-PCR. (c) qRT-PCR was performed to detect the knockdown efficiencies of ALPK2 in the shALPK2 group. (d) The fluorescence expression in cells after 72 h infection was observed. Magnification times: 200x. (e) qRT-PCR was employed for analyzing the expression of ALPK2 mRNA in esophageal cancer cell lines following infection. (f) The expression of ALPK2 protein in esophageal cancer cell lines following infection was detected using western blot. The findings were represented as mean ± SD. ^∗∗^*P* < 0.01 and ^∗^*P* < 0.05.

RETRACTED

**Figure 2:** Depletion of ALPK2 attenuated cell proliferation, migration, and colony formation of esophageal cancer cells. (a) Evaluation of the rate of cell proliferation in esophageal cancer cell lines following infection was determined by the MTT assay. (b) The cell migration rate was detected in esophageal cancer cell lines after being transfected via transwell assay. Magnification times: 200x. (c) The cell migration rate was detected in esophageal cancer cell lines after infection by wound-healing assay. (d) The ability of colony formation was evaluated in esophageal cancer cell lines following infection. The findings were represented as mean ± SD. ^∗∗∗^*P* < 0.001.

**Figure 3:** Depletion of ALPK2 ameliorated cell apoptosis of esophageal cancer cells. (a) Flow cytometry was employed for the determination of the influence of ALPK2 depletion on cell apoptosis. (b) ECL was used to determine the expression of apoptosis-related proteins in TE-1 cells infected with shALPK2 using the Human Apoptosis Antibody Array. Upregulation (*P* < 0.05) was observed for the protein expression as indicated by the results circled in red. (c) Expression of protein was depicted in grayscale, and R studio was used for visualization. (d) The extent of expression of apoptosis-related proteins was analyzed in TE-1 cells with shALPK2. The results were given as mean ± SD. ^∗∗∗^*P* < 0.001, ^∗∗^*P* < 0.01, and ^∗^*P* < 0.05.

**Figure 4:** Depletion of ALPK2 curbed esophageal cancer tumorigenesis. (a) ALPK2 knockdown model based on nude mice was constructed. (b) The evaluation of tumor volume was carried out from feeding to sacrifice. (c) The measurement of the tumor weight was carried out after scarifying the mice. (d) Tumors were photographed following removal. (e) Prior to sacrificing the mice, the intensity of fluorescence was obtained via D-Luciferase injection. (f) The detection of Ki-67 value was carried out in tumor sections using IHC. Magnification times: 200x. (g) Detection of the expression of Akt, P-Akt, mTOR, P-mTOR, CDK6, and PIK3CA was made by western blot. The findings were represented as mean ± SD. ^∗∗^*P* < 0.01 and ^∗∗∗^*P* < 0.001.

**Figure 5:** ALPK2 depletion impaired esophageal cancer development via the downregulation of ITGA11. (a) The coexpressed genes of ALPK2 were predicted via analyzing the Coexpedia website. (b) The levels of PAPPA, ITGA11, and RAB31 were assessed in ESCA samples from TCGA database using the UALCAN website. (c) The association between PAPPA, ITGA11, and RAB31 with ALPK2 was constructed with the ENCORI website. (d) Eca-109 cell proliferation was tested after being transfected with shPAPPA, shITGA11, and shRAB31. The viability and migration of (e) Eca-109 and (f) TE-1 cells were measured in different groups. NC (OE+KD) as negative control; ITGA11+NC-shALPK2 as overexpressed ITGA11; shALPK2+NC-ITGA11 as ALPK2 downregulation; ITGA11+shALPK2 as simultaneously downregulated ALPK2 and overexpressed ITGA11. The findings were represented as mean ± SD. ^∗∗∗^*P* < 0.001, ^∗∗^*P* < 0.01, and ^∗^*P* < 0.05.

RETRACTED

**Table 1:** Patterns of expression of ALPK2 in esophagus cancer tissues and paracarcinoma tissues demonstrated by the immunohistochemistry analysis.

ALPK2 expression	Tumor tissue		Paracarcinoma tissue		*P* value
	Cases	Percentage	Cases	Percentage	
Low	81	51.6%	38	100%	<0.001
High	76	48.4%	—	—	

**Table 2:** Relation between tumor characteristics and ALPK2 expression in individuals with esophagus cancer.

Features	No. of patients	ALPK2 expression		*P* value
		Low	High	
All patients	157	81	76	

Age (years)				0.091
<58	75	44	31	
≥58	82	37	45	
Gender				0.925
Male	111	57	54	
Female	46	24	22	
T infiltrate				0.455
T1	2	1	1	
T2	29	17	12	
T3	86	43	43	
Lymphatic metastasis (N)				0.027
N0	67	41	26	
N1	48	19	29	
N2	2	1	1	
Stage				0.029
I	2	1	1	
II	73	44	29	
III	42	16	26	
Grade				0.634
1	45	23	22	
2	35	17	18	
3	35	20	15	

**Table 3:** Relation between ALPK2 expression and tumor characteristics in individuals with esophagus cancer.

	*N*	ALPK2	
		Spearman correlation	Signification (double-tailed)
Lymphatic metastasis (*N*)	117	0.206	0.026
Stage	117	0.203	0.028

## Data Availability

The data pertaining to the current study can be obtained upon request from the corresponding author.
